# Aberrant Expression TFR1/CD71 in Gastric Cancer Identifies a Novel Potential Prognostic Marker and Therapeutic Target

**DOI:** 10.1155/2022/4257342

**Published:** 2022-08-30

**Authors:** Jielu Cao, Can Hu, Jingli Xu, Jing Han, Ruolan Zhang, Mengxuan Cao, Li Yuan, Zhiyuan Xu

**Affiliations:** ^1^Zhejiang Chinese Medical University, Hangzhou 310053, China; ^2^Department of Gastric Surgery, The Cancer Hospital of the University of Chinese Academy of Sciences (Zhejiang Cancer Hospital), Institutes of Basic Medicine and Cancer (IBMC), Chinese Academy of Sciences, Hangzhou 310022, China; ^3^Key Laboratory of Prevention, Diagnosis, and Therapy of Upper Gastrointestinal Cancer of Zhejiang Province, Hangzhou 310022, China; ^4^Zhejiang Provincial Research Center for Upper Gastrointestinal Tract Cancer, Zhejiang Cancer Hospital, Hangzhou 310022, China

## Abstract

**Background:**

Gastric cancer (GC) is one of the most common malignant tumors with poor prognosis. So far, other than the HER2, GC lacks effective therapeutic targets. Transferrin receptor 1 (TFR1) expressions are abnormally upregulated in various cancers for the satisfaction of iron demand increased. This study aimed to explore the expression and clinical value of TFR1 in GC.

**Methods:**

A tissue microarray including GC tissues and matched noncancerous tissues from 155 GC patients were collected. Moreover, the level of TFR1 expression was detected by immunohistochemistry, and we also evaluated the relationship between TFR1 expression and the clinicopathologic characteristics. What is more, univariate analysis and multivariate analysis were used to evaluate the risk factors and independent risk factors affecting the prognosis of GC.

**Results:**

We found that TFR1 was overexpressed in GC tissues compared with noncancerous tissues, and a significant relationship was found between TFR1 expression and age (*P*=0.001), Lauren type (*P*=0.008), T stage (*P*=0.003), HER2 (*P*=0.003), PD-L1 (*P* < 0.001), and the level of CA72-4 (*P*=0.028). Survival analysis confirmed that GC patients with positive TFR1 expression had a poorer OS than that with negative TFR1 expression, and TFR1 expression was an independent risk factor in GC. Furthermore, we also found that there was a significant difference between the TFR1-PD-L1− group and the TFR1+PD-L1+ group (*P*=0.023), while there was no significant difference between the TFR1-PD-L1− group and the TFR1+PD-L1− group (*P*=0.119), or between the TFR1-PD-L1− group and the TFR1-PD-L1+ group (*P*=0.396).

**Conclusions:**

TFR1 was overexpressed in GC and its aberrant expression identifies a novel potential prognostic marker and therapeutic target. In addition, TFR1 expression may be associated with the immune microenvironment and suppress the immune response via regulating the PD-L1 expression.

## 1. Introduction

Gastric cancer (GC), as a malignant tumor of high invasiveness and heterogeneity, is a critical health problem in the world [1]. Over the past few decades, the incidence of GC has declined in most parts of the world, but the number of new cases still exceeds 1 million each year, and China accounts for nearly half of GC diagnoses each year in the world [2]. Most GC patients are diagnosed at the late stages, because of no symptoms in the early stage. In recent years, targeted therapy and immunotherapy have opened a new field of cancer treatment, but the 5-year overall survival (OS) of GC is still pessimistic. Therefore, finding effective therapeutic targets and markers is necessary for the treatment of GC.

Transferrin receptors (TFRs) are type II membrane glycoproteins, which can import iron to cells by binding transferrin (TF), including transferrin receptor 1 (TFR1) and transferrin receptor 2 (TFR2). TFRs share 66% homology structurally and both consist of two disulfide-linked monomers joined by two disulfide bonds [3]. TFR1 is widely expressed and has a higher affinity for TF, while TFR2 is mostly expressed in hepatocytes and erythroid cells, whereas TFR1 has been found to join in the progression of many tumors, such as brain cancer [4], breast cancer [5], and colon cancer [6]. TFR1, also called cluster of differentiation 71 (CD71), binds to holo-TF to initiate the internalization of the complex by clathrin-mediated endocytosis [7]. TFR1 expressions are abnormally upregulated in various cancer cells for the satisfaction of iron demand increased [8]. Recently many studies have strongly approved that the overexpression of TFR1 links to poor prognosis and the promotion or progression of malignant tumors. Moreover, TFR1 has also been shown to be a potential target for cancer therapy. Yang et al. developed a monoclonal antibody JST-TFR09 against human TFR1, which can interfere with the binding between TFR1 and TF and induce apoptosis in adult T cell leukemia/lymphoma (ATLL) [9]. However, there are few studies on the correlation between TFR1 and GC. In this study, we aimed to evaluate the expression level of TFR1 in GC patients and analyze its impact on the progression and prognosis of GC.

## 2. Methods

### 2.1. Patients and Samples

In this study, 155 patients who underwent surgery were recruited from Zhejiang Cancer Hospital (ZJCH) during the years from January 2013 to December 2017. Meanwhile, we collected demographic information and clinical-pathological characteristics for analyzing the relationship between those variables and TFR1 expression. These patients did not receive antitumor treatments before the operation or suffered from other types of malignant tumors. Formalin‐fixed, paraffin‐embedded (FFPE) GC tissues and adjacent nontumor (NT) tissues that matched these patients were collected to be the samples for immunohistochemistry (IHC). Each tumor pathology diagnosis depended on two pathologists' dependent screening. Standardized chemotherapy was given to patients soon after the operation according to the postoperative pathological results. Regular examination and follow-up were carried out to define overall survival (OS).

### 2.2. Immunohistochemistry (IHC)

The FFPE tissue microarray was constructed with the most representative GC tissues and matched NT tissues and stained in the IHC technique. The FFPE tissue microarray was dewaxed by xylene and rehydrated with graded ethanol. After 3 times of cleaning with 1×PBS on the shaker, 3% hydrogen peroxide was used for antigen repair. We blotted the moisture around the tissue with filter paper. The FFPE tissue microarray was completely covered and sealed with 10% goat serum at room temperature for 20–30 minutes. The FFPE tissue microarray was placed overnight with a primary antibody against TFR1 (ab125066) under a gentle shaker at 4°C that followed. After washing, those were reacted with sheep antirabbit IgG secondary antibody at room temperature for about 30 minutes. 3,3′‐Diaminobenzidine (DAB) was used to observe the antibody binding under a microscope. The nuclei were restained with hematoxylin. The tissue slices were dehydrated with graded ethanol and fixed on a cover glass with a neutral resin.

### 2.3. Evaluation of TFR1 Staining

All IHC results were blindly evaluated by two pathologists. The results of section staining relate to the staining intensity and the percentage of positive staining cells in the region. We used an H-score system to evaluate TFR1 expression in cells. The calculation formula was mentioned as follows: H-score = IS × AP. AP value was assigned according to the proportion of positive staining tumor cells in the field of vision, as follows: 0 (0%), 1 (1%–25%), 2 (26%–50%), 3 (51%–75%), and 4 (75%–100%). The value of IS was determined by the intensity of staining, from 0 to 3 corresponding to no staining, weak staining, medium staining, and strong staining. IHC staining results of at least 3 regions were individually evaluated by each investigator, and H-score was calculated and averaged.

### 2.4. Statistical Analysis

Statistical analysis was conducted using BM SPSS Statistics for Mac, version 25.0 (IBM Corp). A chi-square test was used to analyze the association between TFR1 expression and GC clinicopathological features. The survival curve was drawn using the Kaplan–Meier method. Univariate and multivariate analyses for independent factors of prognosis for patients with GC were conducted using the Cox proportional hazards regression model. A *P* value <0.05 showed statistical significance.

## 3. Results

### 3.1. Patients Characteristics

155 GC patients were collected. Among them, 113 patients were male and 43 patients were female, with a median age of 61 (range 28–86) years. Pathologically, 74 patients were defined as intestinal type, 55 as diffuse type, and 24 as mixed type while 2 were missing information of Lauren type. According to the depth of tumor invasion in the 8^th^ AJCC staging system, 2 patients were in the T1 stage, 6 patients were in the T2 stage, and 13 patients were in the T3 stage, while 134 patients were in the T4 stage. For lymph node metastasis, 10 patients were in the N0 stage, while 145 patients have lymph node metastasis, including 32 patients in the N1 stage, 43 patients in the N2 stage, and 70 patients in the N3 stage. For distant metastasis, 140 patients were in the M0 stage and 15 patients were in the M1 stage. For the TNM stage, 1 patient was in the I stage, 19 patients were in the II stage, and 120 patients were in the III stage, while 15 patients were in the IV stage (as shown in Table 1).

### 3.2. The Expression of TFR1 in GC

TFR1 expression in GC tissues was in dispute. As shown in Table 2 and Figure 1, TFR1 was overexpressed in GC tissues compared with noncancerous tissues. According to H-core, an H-score≥1.0 was defined as a positive TFR1 expression, and an H-score = 0 was defined as a negative TFR1 expression. 197 GC patients showed positive TFR1 expression, while 58 GC patients showed negative expression in GC tissues. However, 64 noncancerous tissues showed positive TFR1 expression, while 91 showed negative TFR1 expression (*P* < 0.001).

### 3.3. The Relationship between TFR1 Expression and Clinicopathological Variables

The chi-square test was used to investigate the association between TFR1 expression and clinicopathological variables in GC. As shown in Table 2, a significant relationship was found among TFR1 expression and age (*P*=0.001), Lauren type (*P*=0.008), T stage (*P*=0.003), HER2 (*P*=0.003), PD-L1 (*P* < 0.001), and the level of CA72-4 (*P*=0.028), while TFR1 expression was not significantly associated with gender, tumor location, Borrmann type, differentiated degree, N stage, and TNM stage.

### 3.4. The Prognostic Value of TFR1 Expression in GC Patients

As shown in Figure 1, we investigated the prognostic value of TFR1 expression in GC. According to K–M plotter databases, the prognostic value of TFR1 expression in GC was in dispute, and the 208691_at cohort and 207332_s_at cohort showed that high TFR1 expression was associated with better prognosis, while the 237215_s_at cohort showed that high TFR1 expression was associated with poorer prognosis. In our study, we found that GC patients with positive TFR1 expression have a better 3-year OS than that with negative TFR1 expression (*P* = 0.012). Moreover, univariate analysis found that tumor location (*P* = 0.045), Lauren type (*P* = 0.045), Borrmann type (*P* = 0.002), N stage (*P* < 0.001), M stage (*P* < 0.001), the level of CEA (*P* < 0.001), the level of CA125 (*P* < 0.001), and TFR1 expression (*P* = 0.018) were the risk factors affecting the prognosis of GC. Furthermore, multivariate analysis found that N stage (*P* = 0.003), M stage (*P* = 0.003), the level of CEA (*P* = 0.010), the level of CA125 (*P* = 0.029), and TFR1 expression (*P* = 0.047) were the independent predictive factors in the OC of GC patients (as shown in Table 3).

### 3.5. The Relationship between TFR1 Expression and PD-L1 Expression or HER2 Expression

Furthermore, according to the expression of TFR1 and PD-L1, all patients were divided into four groups, including negative TFR1 and PD-L1 expression (TFR1-PD-L1−) group, negative TFR1 expression with positive PD-L1 expression (TFR1-PD-L1+) group, positive TFR1 expression with negative PD-L1 expression (TFR1+PD-L1−) group, and positive TFR1 and PD-L1 expression (TFR1+PD-L1+) group. There was a significant difference between the TFR1-PD-L1− group and the TFR1+PD-L1+ group (*P*=0.023), while there was no significant difference between the TFR1-PD-L1− group and the TFR1+PD-L1− group (*P*=0.119), or between the TFR1-PD-L1− group and the TFR1-PD-L1+group (*P*=0.396) (as shown in Figure 2). What is more, according to the expression of TFR1 and HER2, all patients were divided into four groups, including negative TFR1 and HER2 expression (TFR1-HER2−) group, negative TFR1 expression with positive HER2 expression (TFR1-HER2+) group, positive TFR1 expression with negative HER2 expression (TFR1+HER2−) group, and positive TFR1 and HER2 expression (TFR1+HER2+) group. There was a significant difference between the TFR1-HER2− group and the TFR1+HER2− group (*P*=0.010), while there was no significant difference between the TFR1-HER2− group and the TFR1-HER2+ group (*P*=0.469), or between the TFR1-HER2− group and the TFR1+HER2+ group (*P*=0.565) (as shown in Figure 3).

## 4. Discussion

GC is the third most common leading cause of cancer death in the world [10], for it is always diagnosed in the advanced stage and difficult to diagnose in the early stage. Surgery is still the only chance of curing GC, but after curative resection, the recurrence of GC is common [11]. In the advanced stage of GC, drug therapy becomes the main means. However, the efficacy of current traditional chemotherapy is limited and the GC patients' median overall survival is low [12]. So, the analysis of underlying pathogenesis and the research on treatment intervention targets for GC have become the present research hotspot.

In recent years, abnormal iron metabolism has been considered one of the specific markers of tumors. Recent studies have shown that tumors can help themselves gain a growth advantage by altering their iron metabolism [13]. In addition, abnormal iron metabolism, especially iron overload, is closely associated with tumorigenesis and cancer development. The TFR1 is the most important membrane protein regulating iron transport in cells. When cells become cancerous, the process of iron absorption through TFR1 has become one of the most important ways for tumor progression and metastasis. The expression of TFR1 protein in tumor tissues of hepatocellular carcinoma (HCC) patients was found significantly higher than that in adjacent tissues, and the expression of TFR1 in HCC is related to the level of AFP [14]. In addition, with the development of HCC, the expression of TFR1 will be gradually increased. Moreover, a clinical study based on 674 patients with breast cancer showed that high TFR1 expression was strongly associated with poor prognosis in patients [8,15]. Meanwhile, TFR1 expression in benign breast diseases was significantly lower than that in precancerous lesions and invasive cancers, and TFR1 expression in high-grade breast cancer was also significantly higher than that in other grade types of breast cancer [16]. In colon cancer, TFR1 was overexpressed and high expression of TFR1 could activate the IL-6/IL-11-STAT3 signaling pathway and promote the proliferation and apoptosis of colon epithelial cells, thus aggravating the injury of colon mucosa and leading to the occurrence of colon cancer [17]. In our study, we found that TFR1 was overexpressed in GC and the positive rate of TFR1 in GC tissues was higher than that in noncancerous tissues. Moreover, the TFR1 expression was significantly associated with age (*P* = 0.001), Lauren type (*P* = 0.008), T stage (*P* = 0.003), HER2 (*P* = 0.003), PD-L1 (*P* < 0.001), and the level of CA72-4 (*P* = 0.028) in GC. Further analysing, we found that the 3-year OS in TFR1-positive expressed GC was higher than that in TFR1 negative expressed GC. Interestingly, we also found that there was a significant difference between the TFR1-PD-L1− group and the TFR1+PD-L1+ group (*P* = 0.023), while there was no significant difference between the TFR1-PD-L1− group and the TFR1+PD-L1− group (*P* = 0.119), or between the TFR1-PD-L1− group and the TFR1-PD-L1+group. These remind us that TFR1 has relevance to PD-L1. Chen et al. [18]found that TFR1 affected the prognosis of breast cancer patients by regulating the infiltration of immune cells, including CD4+ T cells, CD8+ T cells, B cells, neutrophils, macrophages, and dendritic cells. We suspect that TFR1 expression may be associated with the immune microenvironment and suppress the immune response via regulating the PD-L1 expression. However, the specific regulatory mechanism of TFR1 in GC remains unclear. Shirakihara et al. [19] confirmed that TFR1 will be phosphorylated at tyrosine 20 (Tyr20) in an FGFR2 kinase activity-dependent manner by binding to EGFR2. Moreover, knockdown of TFR1 can block the iron uptake and suppress the cellular proliferation in vitro in diffuse-type GC. However, Cheng et al. [20] confirmed that TFR1 was overexpressed in GC, and TFR1 was negatively correlated with patient prognosis, and its negative TFR1 GC cells were more aggressive. Although TFR1-positive cancer cells can be killed by H-ferritin drug nanocarrier when treated with IFN-*γ*, TFR1-deficient cells can upregulate the expression of PD-L1, CXCL9, and CXCL10 to promote immune escape. This result revealed a different prognostic value of TFR1 expression shown in the present study. We cannot explain this difference because of the different antibodies used to detect the TFR1 expression between the two studies. It is necessary to study the function of TFR1 in regulating GC development, such as immune microenvironment. What is more, we also confirmed that TFR1 expression was an independent prognostic factor for OS in GC patients.

Therefore, TFR1 is expected to be an effective target molecule for tumor therapy. Up to now, as an antihuman TFR1 antibody, JST-TFR09 has a strong affinity with TFR1 in human lymphoma cells and can inhibit iron uptake by interfering with the binding of TFR1 and TF [9]. Moreover, anti-TFR1 monoclonal antibody A24 can significantly inhibit the proliferation and induce apoptosis of malignant cells in T cell leukemia [21]. In addition, the development of nanoscale TFR1-targeting drugs also provides a new direction for the development of TFR1-specific inhibitors in the field of precision-targeted tumor therapy in the future [22].

## 5. Conclusions

TFR1 was overexpressed in GC and its aberrant expression identifies a novel potential prognostic marker and therapeutic target. In addition, TFR1 expression may be associated with the immune microenvironment and suppress the immune response via regulating the PD-L1 expression.

## Figures and Tables

**Figure 1:** TFR1 is overexpressed in gastric cancer tissues. (a) TFR1 expressed in representative tumor tissues and noncancerous tissues in GC. (b) The TFR1 expression was different in tumor and noncancerous tissues (*n*=155). (c) The GC patients with positive TFR1 expression had a better OS than that with negative TFR2 expression. (d–f) The different prognostic value of TFR1 expression in different GC cohort in K–M plotter databases.

**Figure 2:** TFR1 expression was correlated with PD-L1 expression in GC tissues. (a) TFR1 and PD-L1 coexpressed in representative tumor tissues in GC. (b) TFR1 expression was positively correlated with PD-L1 expression (*n*=155). (c) There was a significant difference between the TFR1-PD-L1− group and the TFR1+PD-L1+ group, while there was no significant difference between the TFR1-PD-L1− group and the TFR1+PD-L1− group, or between the TFR1-PD-L1− group and the TFR1-PD-L1+group.

**Figure 3:** TFR1 expression was correlated with HER2 expression in GC tissues. (a) TFR1 and HER2 coexpressed in representative tumor tissues in GC. (b) TFR1 expression was positively correlated with HER2 expression (*n*=155). (c) There was a significant difference between the TFR1-HER2− group and the TFR1+HER2− group, while there was no significant difference between the TFR1-HER2− group and the TFR1-HER2+ group, or between the TFR1-HER2−group and the TFR1+HER2+ group.

**Table 1:** Differential expression of TFR1 in cytoplasm and gastric tissues.

	N	TFR1 expression		Chi-square	*P* value
		Positive	Negative	Value	
Gastric cancer	155	97	58	14.073	<0.001
Noncancerous tissues	155	64	91		

^*∗*^Statistically significant (*p* < 0.05).

**Table 2:** Correlation of TFR1 expression and clinicopathological characteristics.

Variables		TFR1 expression		Total	*X*2	*P* value
		Positive	Negative			
Age (y)						
	≥60	67	25	92	10.146	0.001^*∗*^
	<60	30	33	63		

Gender						
	Male	74	39	113	1.907	0.167
	Female	23	20	43		

Location						
	Proximal	35	13	48	4.413	0.110
	Distal	54	42	96		
	Total	8	3	11		

Lauren type						
	Intestinal type	55	19	74	11.821	0.008^*∗*^
	Diffuse type	28	27	55		
	Mixed type	14	10	24		
	Unknown	0	2	2		

Borrmann type						
	I + II	50	39	89	4.118	0.128
	III + IV	46	18	64		
	Unknown	1	1	2		

Differentiated degree						
	Well/moderate	21	6	27	3.225	0.073
	Moderate-poor/poor	76	52	128		

T stage						
	T1+2	1	7	8	9.035	0.003^*∗*^
	T3+4	96	51	147		

N stage						
	N0+N1	23	19	42	1.504	0.220
	N2+N3	74	39	113		

M stage						
	M0	86	54	140	0.820	0.365
	M1	11	4	15		

TNM stage						
	I + II	9	11	20	3.031	0.082
	III + IV	88	47	135		

HER2						
	Positive	17	1	18	8.830	0.003^*∗*^
	Negative	80	57	137		

PD-L1						
	Positive	46	8	54	18.083	<0.001^*∗*^
	Negative	51	50	101		

CEA						
	Positive	30	10	40	3.551	0.060
	Negative	67	48	115		

CA125						
	Positive	10	3	13	0.668	0.414
	Negative	87	55	142		

CA72-4						
	Positive	24	6	30	4.820	0.028^*∗*^
	Negative	73	52	125		

AFP						
	Positive	8	0	8	3.500	0.061
	Negative	89	58	147		

CA19-9						
	Positive	35	16	51	1.187	0.276
	Negative	62	42	104		

**Table 3:** Prognostic factors in the univariate and multivariate analyses for GC patients.

Parameters	Univariate	Multivariate		
	*P-*value	HR	95% CI	*P-*value
Age	0.575	—	—	—
Gender	0.792	—	—	—
Location	0.045^*∗*^	1.260	0.841–1.889	0.262
Lauren type	0.005^*∗*^	1.289	0.941–1.766	0.114
Borrmann type (I/II vs. III/IV)	0.002^*∗*^	1.343	0.847–2.130	0.209
Differentiated degree (well/moderate vs. moderate-poor/poor)	0.906	—	—	—
T stage (T1+2 vs. T3+4)	0.116	—	—	—
N stage (N0+1 vs. N2+3)	<0.001^*∗*^	3.371	1.517–7.488	0.003^*∗*^
M stage (M0 vs. M+)	<0.001^*∗*^	2.744	1.403–5.369	0.003^*∗*^
TNM stage (I/II vs. III/IV)	0.142	—	—	—
HER2	0.689^*∗*^	—	—	—
PD-L1	0.275^*∗*^	—	—	—
CEA	<0.001^*∗*^	1.913	1.166–3.138	0.010^*∗*^
CA125	<0.001^*∗*^	2.189	1.085–4.415	0.029^*∗*^
CA72-4	0.946	—	—	—
AFP	0.568	—	—	—
CA19-9	0.112	—	—	—
TFR1 expression	0.018	1.726	1.007–2.958	0.047^*∗*^

## Data Availability

The datasets generated during and/or analyzed during the current study are not publicly available due to hospital policy but are available from the corresponding author on reasonable request.
